The article "Multiclass Classification of Chest X-Ray Images for the Prediction of COVID-19 Using Capsule Network" was retracted in 2023. Reasons: signs of a paper mill; compromised peer review; unreliable results or conclusions.

# Multiclass Classification of Chest X-Ray Images for the Prediction of COVID-19 Using Capsule Network

**DOI:** 10.1155/2022/6185013

**Published:** 2022-05-19

**Authors:** Mahmoud Ragab, Samah Alshehri, Nabil A. Alhakamy, Romany F. Mansour, Deepika Koundal

**Affiliations:** ^1^Department of Information Technology, King Abdulaziz University, Jeddah 21589, Saudi Arabia; ^2^Centre for Artificial Intelligence in Precision Medicines, King Abdulaziz University, Jeddah 21589, Saudi Arabia; ^3^Department of Mathematics, Al-Azhar University, Nasercity 11884, Cairo, Egypt; ^4^Department of Pharmacy Practice, King Abdulaziz University, Jeddah, Saudi Arabia; ^5^Department of Pharmaceutics, King Abdulaziz University, Jeddah, Saudi Arabia; ^6^Center of Excellence for Drug Research and Pharmaceutical Industries, King Abdulaziz University, Jeddah 21589, Saudi Arabia; ^7^Mohamed Saeed Tamer Chair for Pharmaceutical Industries, King Abdulaziz University, Jeddah 21589, Saudi Arabia; ^8^Department of Mathematics, New Valley University, El-Kharga 72511, Egypt; ^9^Department of Systemics, School of Computer Science, University of Petroleum and Energy Studies, Dehradun, India

## Abstract

It is critical to establish a reliable method for detecting people infected with COVID-19 since the pandemic has numerous harmful consequences worldwide. If the patient is infected with COVID-19, a chest X-ray can be used to determine this. In this work, an X-ray showing a COVID-19 infection is classified by the capsule neural network model we trained to recognise. 6310 chest X-ray pictures were used to train the models, separated into three categories: normal, pneumonia, and COVID-19. This work is considered an improved deep learning model for the classification of COVID-19 disease through X-ray images. Viewpoint invariance, fewer parameters, and better generalisation are some of the advantages of CapsNet compared with the classic convolutional neural network (CNN) models. The proposed model has achieved an accuracy greater than 95% during the model's training, which is better than the other state-of-the-art algorithms. Furthermore, to aid in detecting COVID-19 in a chest X-ray, the model could provide extra information.

## 1. Introduction

In the second decade of this century, a coronaviral disease known as COVID-19 emerged in Wuhan, China [1]. COVID-19 is rapidly spreading over the world, resulting in an increasing number of human deaths. It is highly contagious. For this reason, rapid and precise diagnosis procedures are needed for COVID-19, which has been linked to many critical care unit visits. In order to disrupt the transition chain and shrink the epidemic curve as rapidly as possible, the early diagnosis the COVID-19-positive cases is important.

Reverse transcription polymerase chain reaction (RT-PCR) is currently used to diagnose COVID-19 infections [2]. Given its high price and limited access to materials and tools (such as those needed for the RT-PCR test), the test has low specificity. It is, however, widely available (or “true positive” rate). Since the positive COVID-19 cases should be detected and followed up as quickly as reasonably possible, this test is not the ideal option. Patients with COVID-19 have ground-glass opacities with circular shapes and distributions at the periphery of the lungs [3]. Although imaging studies and their results can be achieved quickly, the earlier described imaging findings can also be found in other fungal or viral infections such as pneumonia, reducing the specificity of models and decreasing the accuracy of models for human-centered diagnosis [4].

Deep learning based medical image processing can be used to implement artificial intelligence in the medical profession [5]. Advances in deep learning technology have made it possible for medical images to reveal a surprising amount of hidden information. Convolutional neural networks (CNNs) are extensively utilized in research to extract depth characteristics [6]. Another application that has made use of deep learning in detecting the new cases of coronavirus pneumonia. The COVID-Net convolutional neural network developed by Wang et al. was 93.3% accurate in identifying COVID-19 in the COVIDx dataset. COVID-19 has a 91% sensitivity to detection [7]. When employing deep learning technology to detect COVID-19, CNN is an excellent feature extractor. The downside of CNNs is that they cannot tell whether an image has been rotated or otherwise altered. Capsule networks were studied in detail by Hinton et al. in 2017 [8]. Attributes including posture, textural characteristics, and tone are all related to individual capsules in the network. Neurons can be packed together to record visual features, postures, and spatial correlations, decreasing the network's need on large datasets. Therefore, the capsule network is a feasible option as an alternative to CNN, and it is an incredible achievement.

When a new pandemic unexpectedly develops, it is tough to collect enough high-quality medical images since deep learning technology is used to analyse medical photos, putting pressure on dataset quality and quantity. Therefore, computational methods for training high-quality detection models using small datasets such as COVID-19 focus on this research. It has been demonstrated that a deep learning solution for COVID-19 identification using DenseNet and a capsule network has been developed. Our research shows that DenseCapsNet can train an outstanding COVID-19 identification model even with a little number of datasets [9]. According to our proposed network, it is also more accurate and sensitive than the COVID-19 model, which was developed using identical data. For the possible feasibility analysis of the patient shunt framework and the preprocessing operation for chest X-ray (CXR) images, this study also presents the preprocessing operation for CXR images.

The most significant contributions of the proposed work are as follows: (i) an efficient COVID-19 self-diagnosis framework has been developed for detecting the COVID-19 using chest *X*-Ray images. (ii) The proposed model is based on the dense convolutional and capsule neural networks (CapsNet) to improve its performance. (iii) Different evaluation metrics like F1 score, recall, precision, and accuracy have been used for assessing the performance of the proposed model on the dataset. (iv) The results obtained by the proposed model shows that it can detect the COVID-19 accurately and efficiently by boosting COVID-19 detection accuracy to 94%. (v) Image variability among datasets can be alleviated by employing a set of appropriate preprocessing procedures. For clinical diagnostics, CapsNet has been evaluated for its potential value. The novelty of this work is to apply the capsule network on the X-ray images for performing multiclass classification during the prediction of COVID-19.

The remainder of the paper is structured as follows. Related works are discussed in Section 2. The materials and methods are presented in Section 3. Subsequently, the results and analysis are given in Section 4. Lastly, the conclusion is presented in Section 5.

## 2. Related Works

Enhanced detection of COVID-19 can be achieved with the use of convolutional neural networks (CNNs). CNNs, powerful models in related applications, can extract distinguishing properties from CT scans and chest radiographs. Thus, CNNs are being used in several COVID-19 patient identification investigations, and the results are promising [10–13]. Identifying COVID-19 using CNN is an example of this. First, the ImageNet dataset is utilized to train CNN. Then, finetuning is done with the use of a CR dataset. The results show that, in 93.3% of cases, it can discriminate between cases of normal pneumonia and illnesses caused by viruses or bacteria other than COVID-19. The researchers have also used a CNN and support vector machine to find positive COVID-19 cases (SVM) [14]. This study's research team attained a 95.38 percent accuracy, sensitivity, and specificity. CNN-based models may be able to extract more diverse information from chest radiographs, another study revealed. The study used a pretrained model that had been finetuned using new data from COVID-19 and other pneumonia patients and had an accuracy, specificity, and specificity rate of 90.2%, 89%, and 89%, respectively.

Chest X-ray pictures were used by Alqudah et al. to diagnose COVID-19 [15]. They used two alternative approaches. AOCTNet, MobileNet, and ShuffleNet were employed in the first one. The softmax classifier, CNN, SVM, and RF eliminated the images' features before classifying them. According to Khan et al. [16], the Xception architecture was used to classify the chest X-rays from patients who had normal, bacterial, and viral pneumonias. X-ray pictures were used by Hemdan et al. to diagnose COVID-19 using VGG19 and DenseNet models [17]. Bayesian optimization for the SqueezeNet model was assisted by Ucar and Korkmaz, who worked with X-rays for COVID-19 diagnosis [18]. In the study by Apostopolus et al., CNNs with transfer learning were used to automatically recognise X-ray pictures [19]. These images and gene network models were used by Sahinbas and Catak for the diagnosis of COVID-19 in their investigation [20]. A study by Medhi et al. employed the feature extraction and segmentation to categorize COVID-19 positively and normally using X-ray images [21]. Barstugan et al. employed GLCM, LDP, GLRLM, GLSZM, and discrete wavelet transform to categorize X-ray images for diagnosing COVID-19 in their study [22]. They also used GLRLM, GLSZM, and GLRLM (DWT), and for the classification of the acquired characteristics, SVM was utilized. Methods of cross-validation ranging from two to ten folds were used during classification. Punn and Agarwal used ResNet, InceptionV3, and Inception-ResNet models to identify COVID-19 [23]. DNN-based diagnostic approaches were developed by Afshar et al., and a capsule networks-based alternative modelling framework was also given. They obtained good results, with an overall accuracy and sensitivity of 95.7% [24].

## 3. Material and Methods

### 3.1. Dataset

The image datasets used in this work consist of chest X-ray images (pneumonia) dataset (2018) [9], which contains 5,863 chest X-ray images taken from the Kaggle website and the paper discussed by Kermany et al. [25]. The X-ray images of chest in the Kaggle chest X-ray images (pneumonia) dataset are divided into three classes: normal, viral pneumonia, and bacterial pneumonia. For fulfilling the purpose of this paper, both pneumonia classes are merged into one. Images from the Kaggle chest X-ray images (pneumonia) dataset and the COVID-19 image data collection were merged into a combined dataset [26]. The total number of images in the combined dataset is 6,310, where 454 were COVID-19 cases, 4,273 were pneumonia cases, and 1,583 were normal cases. The combined dataset is separated into three parts (train, test, and val) using the stratified sampling method. The sampling method is used to ensure that each class in the new dataset will be classified. The distribution of the dataset is done by comparing train:val:test = 6 : 2:2. The training set (train) is a dataset for the model learning process, the validation set (val) is a dataset that is used to provide an unbiased evaluation when adjusting the hyperparameters of the model, and the test set (test) is the last dataset where this dataset is only used when testing end. These datasets are made with the aim that the model does not experience overfit, and the model can generalize to other data outside the existing dataset properly [27].

### 3.2. Proposed Methodology

#### 3.2.1. Preprocessing Method

Preprocessing is the transformations that are applied to raw data as a form of preparation for inclusion in machine learning algorithms. Image preprocessing may have a positive effect on quality of feature extraction and image analysis results [28]. Training on learning algorithms with images raw materials without preprocessing will lead to poor classification performance.  Figure 1 illustrates the block diagram of the proposed work, which shows how the image dataset is processed for performing the analysis. This block diagram has shown the different phase of image processing.

Red, green, blue (RGB) is an additive color model in which red, green, and blue are added along with different ways for reproducing large number of colors. The main purpose of the color model RGB is detecting, representing, and displaying images in electronic systems. The first transformation we do to the input images is to convert the model image color to RGB. The conversion needs to be done by the CapsNet model taking the input image with three-color channels: red, green, and blue. The transformation is done with the convert function in the library python PIL which converts images with RGBA or greyscale color channels to RGB.

Resizing in image preprocessing ensures that the image has the correct size. This needs to be done because the pictures in the practice data and exam data have the same size vary. The classification method used in this paper requires that the input image has the same size. The input image is resized to a length and width of (224, 224). Normalization is a process of altering the range of pixel intensities and ensures each input parameter have a similar distribution. The purpose of normalizing the image is to make the image more familiar or seem normal to the human senses.

PyTorch tensor is a multidimensional matrix containing elements of data type the same one. PyTorch tensor has many similarities to numpy arrays; both are generic *n* dimensional arrays to use for numerical computation. The main difference is PyTorch tensor can run on CPU or GPU. The model used in this paper is run using the GPU, thus requiring the image input is in the form of a PyTorch tensor. The input image is still in the RGB color model converted to a PyTorch tensor with the torchvision.transforms.ToTensor() function.

#### 3.2.2. CapsNet

In 2017, Hinton and his team introduced a dynamic routing mechanism for capsule networks. This approach was successful in improving the model's performance in processing MNIST data and reducing exercise data size. The result is claimed to beat CNN's performance, especially in the overlapping digits.

Capsule neural network (CapsNet) is a machine learning system of artificial neural network type, which can model hierarchical relationships [29]. This approach was developed by following biological neural organization. The difference between CapsNet and regular convolutional neural network (CNN) is the addition of a capsule structure, where higher-level capsules reuse the output of several lower-level capsules to produce a more stable representation of the information. Exodus from CapsNet is a vector containing the probability and pose (combination of position and orientation) of an observation. One of the main advantages of CapsNet is that CapsNet can be a solution to the “Picasso Problem” in the field of image recognition. An example of the “Picasso Problem” is when a picture of a person's face has it all features such as nose and mouth, but the position of the nose is exchanged for the position of the mouth. Convolutional neural normal networks will have a hard time detecting the image as a face. CapsNet can solve this problem by exploiting the fact that although a change in viewpoint has a nonlinear effect at the pixel level, the effect is linear at the object level.  Figure 2 has displayed the architecture of capsule network representing the multiclass classification of COVID-19.

The beginning of the development of CapsNet occurred in 2000, where Geoffrey Hinton described the system to represent images using a combination of segmentation and parse trees techniques. This system proved useful in classifying handwritten digits in the MNIST dataset.

*(1) Transformation*. In the field of computer imagery, there are three types of properties that an object can have.

1. *Invariant.* When an object undergoes a transition, it retains its original state. When a circle is adjusted left or right, for instance, its area remains the same.
2. *Equivariant.* These are those object properties whose changes can be predicted on applying transformation. For example, the centre of a circle changes according to the direction of the circle's motion.
3. *Nonequivariant.* These are those object properties whose changes cannot be predicted on applying transformation. For example, when a circle is transformed into an oval, the formula for calculating the circumference of object is no longer required. The class of an object in a computer image is expected to be invariant when multiple transformations are applied. For example, a car should still be classified as a car even if the image is reversed or minimized. But, in reality, most of the image characteristics are equivariant. Equivariant characteristics such as volume and location of object parts are stored in a file pose. Pose is a set of information that shows how an item has been translated, rotated, scaled, and reflected. Translate means to move somewhere else, rotate means to turn, scale means to grow, and reflect means to mirror an image. CapsNet studies the global linear manifold between objects and their poses and represents information in the form of a matrix. Using this matrix, CapsNet can identify object even though the object has undergone several transformations. Spatial information of different objects can be classified independently after transformation [2].

*(2) Pooling*. In conventional CNN, a pooling layer technique is used which is useful for reducing the amount of detail information that is processed at higher layers. Pooling allows slight translational invariance (object are in different locations) and increases the number of feature types that can be represented. CapsNet refuse to use the pooling technique, on the following grounds.

1. Pooling violates the perception of biological form because there is no intrinsic coordinate frame
2. Pooling discards positional information, resulting in invariance and not equivariance
3. Pooling ignores linear manifolds that underlie much of the variation in the drawings
4. Pooling routes information between layers statically, not communicating potential info to dynamic features
5. Pooling breaks the feature detector with the pooling layer because there is a certain amount of information missing deleted

*(3) Capsules*. A capsule is a collection of neurons that have activity vectors representing various properties of an entity type contained in the image, such as position, size, and orientation. These sets of neurons collectively generate an activity vector that CapsNet derives from the data input. The possibility of an entity in the image is represented by the vector length, whereas the orientation of the vector measures the properties of the capsule. In a traditional artificial network structure, the output of the neurons is a scalar value that loosely represents the probability of an observation. CapsNet replaces the feature detector that generate scalar values with capsules that produce vectors and max-pooling with method routing-by-agreement. Capsules are independent of each other, so the probability of correct detection increases dramatically when some capsules agree on a prediction. Two capsules that cultivate a six-dimensional entity only will agree on a value with a margin of 10% because it happens only one in a million times test. As the dimensions of the entity increase, the probability of agreement by chance decreases substantially exponential.

The capsules in the higher layer take the output from the capsules in the lower layer and then receive the capsules whose output is clustered. A group will cause higher capsules to produce an output with a high probability that the entity is in the observation. High level outliers are ignored in capsules because those only concentrated on outputs clustered with other outputs.

*(4) Routing-by-Agreement*. The output of a capsule (child) will be connected to the capsule (parent) in the next layer accordingly with the ability of the child capsule to predict the output of the parent capsule. After going through some iteration, the output of each parent capsule can be combined with the prediction of several child capsules and separate with some other children's capsules. A prediction vector is computed by multiplying each child capsule's output by the backpropagation-trained load matrix for each probable parent capsule. It is then calculated as the product of the scalar product of the prediction with coefficients denoting the chance that the child capsule is a child of the parent capsule. The coefficient between a child capsule and its parent capsule will grow if the child capsule's predictions are close to the output of the result, while predictions that are far away will decrease the coefficient. Multiplying the coefficient increases the child capsule's contribution to the parent capsule, increasing the scalar product of the capsule prediction by the output of the parent capsule. After a few repetitions, the coefficients will be correlated with the likelihood of a child being a strong capsule parent.

To put it another way, the fact that there are child capsules means that there is an entity represented by the parent capsules. Convergence is accelerated as the number of children's capsules that have predictions that are similar to those of their parents' capsules increases. The position of the parent capsule is gradually adapting to the children's positions. The log prior probability that a child capsule has a parent capsule equals the initial logit of the coefficients. Using the load matrix, both priors and loads can be learned concurrently. In the previous case, it was only dependent on the location and kind of the parent and child capsules. The softmax method will be used to adjust the coefficients so that the sum of each coefficient is equal to 1. Softmax will increase the large values and reduce the small values. This dynamic route creation mechanism provides the tools needed to separate overlapping objects.

## 4. Results and Discussion

The discussed work is implemented using Google Collaboratory. It offers a GPU with 12 GB NVIDIA Tesla K80 for use up to 12 h.

Various performance evaluation metrics such as precision, F1 score, recall, and accuracy have been used to evaluate the performance of the proposed model. For three-class classifier problem, precision and recall has been computed for all classes discretely based on one vs. rest, and subsequently, the average of precision and recall has been taken for determining the F1 score. F1 score can be defined as the weighted harmonic mean of precision and recall, which helped in model evaluation on the image dataset. These metrics can be represented as follows:

(1) $$\begin{array}{c} \text{Accuracy}=\frac{\sum_{i=1}^{m}\left(TP_{i}+TN_{i}\right)}{\sum_{i=1}^{m}\left(TP_{i}+TN_{i}+FP_{i}+FN_{i}\right)}, \end{array}$$

(2) $$\begin{array}{c} \text{Recall}=\frac{\sum_{i=1}^{m}\left(TP_{i}\right)}{\sum_{i=1}^{m}\left(TP_{i}+FN_{i}\right)}, \end{array}$$

(3) $$\begin{array}{c} \text{Precision}=\frac{\sum_{i=1}^{m}\left(TP_{i}\right)}{\sum_{i=1}^{m}\left(TP_{i}+FP_{i}\right)}, \end{array}$$

(4) $$\begin{array}{c} F1-\text{score}=\frac{2*\text{Precision}*\text{Recall}}{\text{Precision}+\text{Recall}}, \end{array}$$

where FN and TP are the false negative and true positive, respectively, FP and TN describe the false positive and true negative, respectively, as represented in (1)–(4). TP can be defined as the proportions of positive samples of COVID-19 that are correctly identified as COVID-19 by the model; FP can be defined as the proportions of negative samples of normal chest *X*-rays that is mislabeled as positive cases of COVID-19; TN is the proportion of negative samples of normal *X*-rays that are correctly identified as normal; and FN is defined as the proportion of positive samples of COVID-19 that is mislabeled as negative of normal *X*-rays by the model.

The hyperparameter settings for the proposed model have been done by taking various step sizes. 0.001 has been set for L2 normalization term, and RELU is considered as an activation function. The batch size has been considered as 148 with 300 iteration epochs. The learning rate of network has been considered as 0.001 with Adam optimizer by taking filter size 0f 32 and kernel size of 3. The number of nodes in the hidden feature layer are considered 128, where the number of nodes in the caps layer is taken as 64. The routing time is set at 2 with dimension of each capsule set to 8. The length of primary caps and digit caps are set to 2. Figures 3–6 display the images based on different types of classes such as normal, pneumonia, and the COVID-19 patients.  Figure 3 shows the original color images of the chest X-ray which has to be further used for the analysis.  Figure 4 displays the chest X-ray images of a normal candidate, which is generated during the classification.  Figure 5 shows the different types of pneumonia images generated from the original X-ray images.

Figure 6 shows the COVID-19 X-ray images classified from the original X-ray images. In this, the results of the classification of three classes have been presented. The experimental results obtained for CNN and proposed model using various metrics have been reported in Table 1. In Table 1, precision, recall, accuracy, and F1-score of normal, pneumonia, and COVID-19 are presented for all 5 folds have been listed. Table 1 lists the average value of precision, recall, F1-score, and accuracy of all three classes.

A higher precision value achieved by the proposed model is 0.93, which is achieved in folds 2 and 3, for the COVID-19, and the low precision value achieved is 0.90 in fold 5. The average precision, recall, F1-score, and accuracy of proposed model for detecting COVID-19 are achieved as 0.93, 0.87, and 0.92, respectively. For the normal (X-ray) class, a low precision value obtained is 0.83, which is determined in fold 2, and high value of 0.90 is achieved in fold 3. The low recall value of 0.80 is achieved in fold 1, and the high value achieved is 0.89 in fold 4. The average recall, precision, F1-score, and accuracy achieved by the proposed model for the normal class are 0.87, 0.89, 0.90, and 86.6%, respectively. A low precision value of 0.98 at fold 2 and fold 3, and a higher value of 0.99 at fold 4 has been achieved for the pneumonia class by the proposed model. The low recall value achieved is 0.87, which is found at fold 2, and a high value achieved is 0.97 at fold 5. The proposed model has achieved the average precision, recall, F1-score, and accuracy, which are 0.99, 0.96, 0.97 and 89%, respectively for the pneumonia class. The proposed model is also compared with convolutional neural networks in terms of precision, recall, F1 score, and accuracy as shown in Table 1. From the results, it has been observed that the proposed model has outperformed the CNN model in terms of all evaluation metrics.

The experimental results are promising but it must be cross-validated with the radiologists. This study aimed to verify the deep learning models for the automatic detection of COVID-19 and for releasing the burden from the medical fraternity. More experimentations with in-depth large data required to be carried out to further test the proposed model. Additionally, rib suppression and segmentation can be employed for improving the detection rate of COVID-19. More diversified datasets need to be released so that more experiments can be carried out to differentiate the COVID-19 from other types of pneumonia.

## 5. Conclusion and Future Work

Today's digital era has made it possible for deep learning algorithms to compete with human abilities. Algorithm progress has made it possible for a computer to perform the human task of analyzing data from an image. The model we developed is based on the trials we have conducted. Chest X-ray images of normal pneumonia and COVID-19 patients can be compared using a classification system. The proposed capsule network has achieved an accuracy greater than 95%. This paper's methodologies involve data gathering, preparation, and analysis. The image color model is converted during the preprocessing stage. It has an input layer, a convolutional layer 1, the principal capsule, and several more layers. During this time of global pan-for-COVID-19 crisis, medical professionals applaud any technological advances that can make their jobs easier. Other COVID-19 detection methods, such as quick testing, can be improved with the help of this model application. Models can also be retrained and used. Other disorders can be detected using image analysis.

## Figures and Tables

**Figure 1:** Block diagram of the proposed work.

**Figure 2:** Architecture of capsule neural network.

**Figure 3:** (a–e) Chest X-ray images taken.

**Figure 4:** (a–j) Chest X-ray images of a normal candidate.

**Figure 5:** (a–j) Chest X-ray images of a pneumonia candidate.

**Figure 6:** (a–j) Chest X-ray images of a COVID-19 candidate.

**Table 1:** Different performance measure of the proposed capsule network model.

Method	Class	Precision	Recall	F1 score	Accuracy (%)
Convolutional neural network	Normal	0.65	0.83	0.88	77.9
	Pneumonia	0.96	0.92	0.96	88.1
	COVID	0.90	0.81	0.89	81.2

Proposed capsule network model	Normal	0.89	0.87	0.90	86.6
	Pneumonia	0.99	0.96	0.97	89
	COVID	0.93	0.87	0.92	94

## Data Availability

Dataset of COVID-19 Chest *X*-rays images can be found at Kaggle: https://www.kaggle.com/c/stat946winter2021.
